# A Nomogram to Predict Noninflammatory Skin Involvement of Invasive Breast Cancer

**DOI:** 10.1155/2022/1823770

**Published:** 2022-06-30

**Authors:** Xueli Zhu, Shaolin Tian, Ran Jiang, Dan Gao, Bo Chen, Wenliang Lu

**Affiliations:** Department of Thyroid and Breast Surgery, Maternal and Child Health Hospital of Hubei Province, Tongji Medical College, Huazhong University of Science and Technology, 430070, China

## Abstract

**Purpose:**

The aim of this study was to develop and assess a nomogram to predict noninflammatory skin involvement of invasive breast cancer.

**Methods:**

We developed a prediction model based on SEER database, a training dataset of 89202 patients from January 2010 to December 2016. Multivariable logistic regression analysis was applied to build a predicting model incorporating the feature selected in the least absolute shrinkage and selection operator regression model. Discrimination, calibration, and clinical usefulness of the predicting model were assessed using the C-index, calibration plot, and decision curve analysis. Internal validation was assessed using the bootstrapping validation.

**Results:**

Predictors contained in the prediction nomogram included use of age, race, grade, tumor size, stage-N, ER status, PR status, and Her-2 status. The model shows good discrimination with a C-index of 0.857 (95% confidence interval: 0.807–0.907) and good calibration. High C-index value of 0.847 could still be reached in the internal validation.

**Conclusion:**

This study constructed a novel nomogram with accuracy to help clinicians access the risk of noninflammatory skin involvement by tumor. The assessment of clinicopathologic factors can predict the individual probability of skin involvement and provide assistance to the clinical decision-making.

## 1. Introduction

International Agency for Research on Cancer (IARC) released the latest global cancer burden data in 2020. The number of new cases of breast cancer in the world ranked first. It is gratifying that the five-year survival rate of breast cancer was nearly 90% in developed countries and 83% in China. More and more surgeons and patients have requirements for postoperative reconstruction of breast cancer surgery (BCS). Over the years, surgical techniques for breast cancer have evolved from mastectomy to breast-conserving surgery and breast reconstruction. Mastectomy [1] including radical mastectomy, or traditional non-skin-sparing mastectomy (NSSM) and skin-sparing mastectomy (SSM), plays an important role in breast surgery. Radical mastectomy remains most commonly performed today and was described by Madden in 1965, which requires removal of varying degrees of skin (NSSM). In contrast with radical mastectomy, SSM requires the preservation of the maximum skin, even overall skin. The skin-sparing mastectomy (SSM) techniques described as entails excision of the biopsy scar, all breast parenchyma, skin overlying a superficial tumor, was first introduced in 1991 by Toth and Lappert [2]. However, whether to remove the skin from the overlying tumor is not accepted by all surgeons [3]. In addition, several meta-analyses showed no significant difference between SSM and non-SSM in oncological considerations [4]. Be that as it may, negative surgical margins are imperative for SSM [5]. Previous retrospective studies have found local recurrence rates of 0.6%-10.4% in SSM and 1.3%-11.5% after mastectomy [6]. A British study found that compared with mastectomy, patients with negative axillary lymph nodes had a 5-fold higher risk of local recurrence after SSM (*P* 0.033) [7]. This means that surgeons need to be cautious when choosing SSM. Once the skin invasion is detected, the skin overlying the tumor cannot be preserved. Generally speaking, clinicians can find the breast skin invasion visually, such as orange peel sign and dimples. Ultrasound, mammography, and MRI can also be used to assess skin involvement. These imaging modalities predict the possibility of skin invasion though measuring the distance between the mass and the skin. Nevertheless, such predictions are inaccurate leading a high false positive rate, simultaneously adding the extra financial burden to patients. Due to limitations of these methods, the skin of breast will be removed more or less.

Despite the shortcomings above, there is currently no model that can directly predict noninflammatory skin involvement so far. Until now, majority of the literature has simply speculated on the tumor safety based on local recurrence or pathological examination, which was definitely lagging behind. In an attempt to fill this vacancy, the research was to establish a nomogram that can directly predict whether the skin of breast cancer patient has been involved or not by mining the SEER database.

## 2. Materials and Methods

### 2.1. Patients

SEER database (https://seer.cancer.gov/) is supported by the Surveillance Research Program of Cancer Control and Population Sciences. Data were extracted from 18 registries within the SEER database from January 2010 to December 2016, which represents approximately 28% of the U.S. population. We only collected critical data available. The following data included age, race, grade, tumor size, stage-N, ER status, PR status, Her-2 status, and molecular subtyping.

Inclusion criteria are as follows: the inclusion patients were all nonmetastatic invasive breast cancers with T1-3 and T4a-T4b tumor staging in AJCC seventh edition, in which T4b was defined as ulceration and/or ipsilateral satellite nodules and/or edema (including peau d'orange) of the skin, which does not meet the criteria for inflammatory carcinoma in AJCC seventh edition.

Exclusion criteria are as follows: (1) unknown distant metastasis; (2) unknown race or grades; (3) unknown ER status, PR status, Her-2 status, or stage N; and (4) nonmetastatic invasive breast cancers with Tx, T0, Tis, T4c, T4d, or T4NOS.

### 2.2. Statistical Analysis

All the patients met the requirements and were enrolled in the primary cohort, which was further randomized into training cohort and validation cohorts following the ratio of 1 : 1 using R, version 3.6.0 (http://www.rproject.org/) (Figure 1).Baseline clinicopathologic characteristics of the patients included were conducted with a descriptive analysis. We utilized the least absolute shrinkage and selection operator (LASSO) method to select the optimal predictive characteristics in risk of noninflammatory skin involvement from the patients with invasive breast cancer; the method is suitable for the reduction in high dimensional data.

We selected characteristics with nonzero coefficients in the LASSO regression model. The characteristics selected from the LASSO regression model were used for multivariable logistic regression analysis to build a model for predicting. In the multivariate logistic regression model, bilateral *P* values < 0.05 were considered to be statistically significant. All the factors with *P* values < 0.05 in multivariate regression were incorporated into the construction of the prediction model.

Then, we used calibration plots to assess the accuracy of nomogram. In order to quantify nomogram's discriminative ability to identify the noninflammatory skin involvement, the Harrell's concordance index (C-index) was performed. R (version 3.6.0) (http://www.r-project.org/) was performed in all statistical analyses. We used the “rms” package in R to build the nomograms.

## 3. Results and Discussion

### 3.1. Patients' Characteristics

A total of 176418 patients eventually enrolled in the study from the SEER database. In the training cohort, noninflammatory skin involvement occurred in 1.2% of invasive breast cancers in the study, which was accordant with the validation cohort. The patients were divided into the training cohort and the validation cohort, and all clinicopathologic features are summarized in Table 1. Of all the clinicopathologic characteristics, eight potential predictors on the basis of 176418 patients in the cohort had nonzero coefficients in the LASSO regression model (see in Table 2 and Figures 2(a) and 2(b)). We performed univariate unadjusted logistic regression analysis to the variables age, race, grade, stage-N, ER status, PR status, Her-2 status, tumor size, and molecular subtyping.

### 3.2. Development of a Nomogram

A nomogram was constructed with the data of training cohort. And significant factors in the logistic regression were used to construct a nomogram. These factors include age, race, grade, stage-N, ER status, PR status, Her-2 status, tumor size, and molecular subtyping (Figure 3). Each factor used to construct the nomogram was assigned a score. By adding these scores, we can predict the possibility of noninflammatory skin involvement of breast cancer patient.

### 3.3. Calibration and Validation of the Nomogram

The C-index of the prediction model was 0.872 in the training group and 0.878 in the validation cohort, respectively, which indicated that the model had good discrimination. The calibration plots showed excellent agreement with both of the training cohort and validation cohort (Figure 4). The ROC curve showed that AUC was 0.868, which indicated that the model had good predictive ability (Figure 5).

## 4. Discussion

At present, whether the patient's skin of breast is invaded is a key issue that both doctors and patients are concerned about when preparing for breast cancer surgery, especially in SSM and BCS. Preoperative evaluation is conducive to the smooth implementation of the surgical process. Further, adequate preoperative assessment can facilitate surgery to achieve the desired results. To achieve these goals, predictive models need to build for clinical decision-making urgently. Nomograms are widely used for tumor-related prediction, which can reduce statistical predictive models into a single numerical estimate of the probability of an event [7]. These user-friendly graphical interfaces can be utilized for facilitating clinical decision-making. Nevertheless, no study has been reported previously about tumor noninflammatory skin involvement. As a consequence, we build a predictive model of noninflammatory skin involvement in invasive breast cancer for the first time and hope to provide clinical reference when making decisions.

In this study, 176481 patients with invasive breast cancer were included from the SEER database in which noninflammatory skin involvement rate was 1.2%, which was in concordance with previous study. Lookingbill et al. [8] analyzed 7,316 breast cancer patients and found that skin involvement was 1.3%. These data show that the probability of skin invasion in breast cancer patients is relatively low. According to principle of oncology, the skin must be essentially removed if the skin has been involved regardless of any procedures. Thus, whether the skin is involved by tumor or not is extremely important. Generally speaking, breast skin involvement is assessed by physical examination and ultrasound, mammography, or MR. M A EL-Adalany et al. analyzed 125 breast cancer patients and found that abnormal unilateral nipple enhancement was the most important independent MRI predictor of malignant NAC invasion (*P* < 0.001) [9]. In this nomogram, we found that age, histological grade, and numbers of lymph node metastases, race, ER status, PR status, Her-2 status, and tumor size were independent predictors of breast cancer skin involvement. Among these factors, histological grade, number of lymph node metastases, and tumor size were strongly correlated with skin involvement. From the perspective of single factor (Figure 3), it was found that the higher the histological grade of breast cancer, the larger the tumor; the more lymphatic metastasis, then the more likely of skin invasion. ER/PR negative, HER-2 positive, and black patients were the high risk factors for skin involvement. It is worth mentioning that women over 50 were more likely to have skin invasion, in which tumor size had the greatest influence.X. M. Yang et al. [10] found that breast cancer patients with larger primary tumor and more regional lymph node metastasis were more likely to have skin invasion. A study found that tumor type, HER-2 status, and PR status were significant predictors of malignant papillary areola complex invasion, and the *P* values are, respectively, 0.006, <0.001, and 0.014 [9]. A British study found that more than 4 lymph node metastases in breast cancer patients (HR 8.0, *P* < 0.001) and involved surgical margins (HR 3.3, *P* = 0.002) were predictor of local recurrence of breast cancer [11]. Obviously, these factors are also traditional risk factors for tumor recurrence, which have been proven in many studies [12, 13]. Güth et al. also observed that patients with a higher number of involved axillary lymph nodes and extensive lymph nodes involvement were more likely to invade the skin of breast [14]. And the results of these studies are similar to our results. A Japanese study recommended to remove the skin covering the tumor at a distance of less than 2 mm from the tumor to the dermis on ultrasound when performed NSM or SSM in invasive breast cancer [15]. In this study, ultrasound was used for evaluation, which was single and subjective. The combination of clinicopathologic data in our study seems to be more convincing.

SEER database represents nearly one-third of the U.S. population. Therefore, the nomogram based on SEER database can be used as a relatively accurate prediction tool to predict noninflammatory skin involvement. In particular, in this study, the C-index of the training cohort and validation cohort was higher, respectively, which can more precisely predict the large sample data. In addition, good discrimination and calibration power were demonstrated in internal validation. A similar conclusion with ROC curve was obtained, which proves that our model has high prediction accuracy.

The skin overlap the tumor plays an important role in numerous breast cancer surgery, especially in breast-conserving surgery, total mastectomy and oncoplastic surgery. In breast-conserving surgery, skin excision may lead to the deviation of the nipple and areola and the asymmetry of bilateral nipple position. In total mastectomy, extra skin flap transplantation may be needed because of the large area cutaneous deficiency in the surgical area. In oncoplastic surgery, skin removal may result in excessive skin tension, implant exposure, and the risk of infection [16, 17]. The nomogram developed in this study can help clinicians predict skin invasion of tumor and then may preserve as much as possible breast skin for patients especially during oncoplastic surgery.

## 5. Conclusions

In conclusion, this study construct a novel nomogram to help clinicians access the risk of noninflammatory skin involvement by tumor. The assessment of clinicopathologic factors can predict the individual probability of skin involvement and provide assistance to the clinical decision-making. In the future, we will verify it further.

## Figures and Tables

**Figure 1:** Data filtering process.

**Figure 2:** Demographic and clinical feature selection using the LASSO binary logistic regression model. (a) Optimal parameter (lambda) selection in the LASSO model used fivefold cross-validation via minimum criteria. The partial likelihood deviance (binomial deviance) curve was plotted versus log (lambda). Dotted vertical lines were drawn at the optimal values by using the minimum criteria and the 1 SE of the minimum criteria (the 1-SE criteria). (b) LASSO coefficient profiles of the 9 features. A coefficient profile plot was produced against the log (lambda) sequence. Vertical line was drawn at the value selected using fivefold cross-validation, where optimal lambda resulted in 8 features with nonzero coefficients. LASSO: least absolute shrinkage and selection operator; SE: standard error.

**Figure 3:** Developed a nomogram. Note: the noninflammatory skin involvement nomogram was developed in the cohort, with the use of age, race, grade, tumor size, stage-N, ER status, PR status, and Her-2 status.

**Figure 4:** Calibration curves of the noninflammatory skin involvement nomogram prediction in the cohort. Note: the *x*-axis represents the predicted medication noninflammatory skin involvement risk. The *y*-axis represents the actual diagnosed noninflammatory skin involvement. The diagonal dotted line represents a perfect prediction by an ideal model. The solid line represents the performance of the nomogram, of which a closer fit to the diagonal dotted line represents a better prediction.

**Figure 5:** ROC curves of the noninflammatory skin involvement nomogram prediction in the cohort. Note: the *x*-axis represents false positive rate of the model. The *y*-axis represents the true positive rate of the model.

**Table 1:** Differences between demographic and clinical characteristics of skin involvement and no skin involvement groups.

Variables	No skin involvement *N* = 174229		Skin involvement *N* = 2189		Total *N* = 176418	
	No.	%	No.	%	No.	%
Year (age)						
<35	3084	1.7	47	2.1	3131	1.7
35-50	30631	18.1	310	14.1	30941	18.1
>50	140514	80.0	2832	83.0	143346	80.1
Race						
White	138310	79.3	1596	72.9	139906	79.3
Black	15990	9.1	359	16.4	16349	9.2
Other	19929	11.4	234	10.6	20163	11.4
Grade						
I	44395	25.4	149	6.8	44544	25.2
II	72135	44.8	812	37.0	78947	44.7
III	51293	29.4	1210	55.2	52503	29.7
IV	406	0.2	18	0.8	424	0.2
Stage_N						
N0	125776	72.1	584	26.6	126360	71.6
N1	36850	21.1	884	40.5	37737	21.3
N2	7629	4.3	401	18.3	8030	4.5
N3	3974	2.2	317	14.4	4291	2.4
ER						
Positive	148492	85.2	1583	72.3	150075	85.0
Negative	25737	14.7	606	27.6	26343	14.9
PR						
Positive	129851	74.5	1291	58.9	1331142	74.3
Negative	44378	25.4	898	41.0	45276	25.6
Her-2						
Positive	22689	13.0	525	23.9	23214	13.1
Negative	151540	86.9	1664	76.0	153204	86.8
Size (cm)						
≤2	110598	63.4	218	10.4	110816	62.8
2-5	53596	30.7	918	41.9	54514	30.9
> 5	10035	5.7	1043	47.6	11078	6.2
Subtype						
Luminal A	133071	76.3	1281	58.5	134352	76.1
Luminal B	17014	9.7	334	15.2	17384	9.8
HER-2 rich	5675	3.2	191	8.7	5866	3.3
Triple negative	18469	10.6	383	17.4	18852	10.6

ER: estrogen receptor; PR: progesterone receptor; HER2: human epidermal growth factor receptor 2; Grade: histological grade.

**Table 2:** Prediction factors for noninflammatory skin involvement.

Variable	*β*	OR (95% CI)	*P* value
Age			
>50		1	
35-50	0.01559548	0.448640 (0.3960100-0.50826)	≤0.001
<35	0.81713909	0.441690 (0.3960100-0.50826)	≤0.001
Race			
White		1	
Black	0.32953753	1.390300 (1.2310000-1.57030)	≤0.001
Other	0.03695001	1.037600 (1.02996900-1.19680)	≤0.001
Grade			
II		1	
I	0.48567067	0.615280 (0.5141500-0.73631)	≤0.001
III	0.83569417	1.419100 (1.2822000-1.57060)	≤0.001
IV	1.33994164	2.349700 (1.4125000-3.90860)	≤0.001
Stage_N			
N-N0		1	
N-N1	0.90441662	2.470500 (2.2110000-2.76050)	≤0.001
N-N2	1.27886054	3.592500 (3.1285000-4.12540)	≤0.001
N-N3	1.41222087	4.105100 (3.5259000-4.77930)	≤0.001
ER			
Positive		1	
Negative	0.13946618	1.149700 (1.0034000-1.31730)	0.003
PR			
Positive		1	
Negative	0.07585678	1.0788000 (1.0049600-1.21870)	0.005
Her_2			
Negative		1	
Positive	-0.29043028	1.337000 (1.2027000-1.48630)	≤0.001
Size			
≤2 cm		1	
2-5 cm	1.61425616	5.024100 (4.3187000-5.84480)	≤0.001
> 5	3.18112184	24.074000 (20.5890000-28.14800)	≤0.001

Note: *β* is the regression coefficient.

## Data Availability

The study data are from SEER database (https://seer.cancer.gov/).
